This article has been retracted.

# MicroRNA-625 inhibits cell invasion and epithelial–mesenchymal transition by targeting SOX4 in laryngeal squamous cell carcinoma

**DOI:** 10.1042/BSR20181882

**Published:** 2019-01-22

**Authors:** Yuan Li, Chenjuan Tao, Lili Dai, Caixia Cui, Chaohui Chen, Honglin Wu, Qingyu Wei, Xuehua Zhou

**Affiliations:** 1 Department of Otolaryngology Head and Neck Surgery, Affiliated Hospital of Hangzhou Normal University, Hangzhou 310015, China; 2 Department of Neurology, Affiliated Hospital of Hangzhou Normal University, Hangzhou 310015, China

**Keywords:** epithelial-mesenchymal transition, laryngeal squamous cell carcinoma, microRNA-625, SOX4

## Abstract

Introduction: Laryngeal squamous cell carcinoma (LSCC) is a highly aggressive malignant cancer, but the molecular mechanisms underlying its development and progression remain largely elusive. The purpose of the present study is to investigate the expression profile and functional role of microRNA-625 (miR-625) in LSCC.

Materials and methods: LSCC tissues and adjacent normal tissues were collected from 86 LSCC patients. The expression levels of miR-625 and SOX4 mRNA in tissues and cells were detected by RT-qPCR analysis. The expression levels of SOX4 and EMT-related proteins were detected by western blot analysis. *In vitro* cell proliferation, migration, and invasion were detected by MTT assay, colony formation assay, wound healing assay, and transwell invasion assay, respectively. Dual-luciferase reporter assay was performed to verify the binding relationship between miR-625 and the 3′-UTR of SOX4.

Results: The results demonstrated that miR-625 is significantly down-regulated in clinical LSCC tissues, and its low expression may be closely associated with unfavorable clinicopathological characteristics of LSCC patients. Overexpression of miR-625 significantly suppressed the proliferation, migration, invasion, and EMT of LSCC cells. Furthermore, SOX4 was validated as a direct target of miR-625 in LSCC cells, and rescue experiments suggested that restoration of SOX4 blocked the tumor suppressive role of miR-625 in LSCC cells.

Conclusions: Taken together, these findings highlighted a critical role of miR-625 in the pathogenesis of LSCC, and restoration of miR-625 could be considered as a potential therapeutic strategy against this fatal disease.

## Introduction

Laryngeal cancer is one of the most common head and neck cancers, and laryngeal squamous cell carcinoma (LSCC) accounts for approximately 85–90% of all laryngeal cancer cases [1]. In spite of recent advances in diagnostic and therapeutic methods, the long-term prognosis of LSCC patients remains largely unsatisfactory [2]. Accordingly, a complete understanding of the molecular mechanisms that are involved in LSCC development and progression is of critical importance.

MicroRNAs (miRNAs), initially identified in 1993, are a class of endogenous small (∼22 nucleotide) noncoding RNAs that play critical regulatory roles in animals and plants by targeting mRNAs for cleavage or translational repression [3,4]. A growing body of evidence indicates that miRNAs can function as potential oncogenes or tumor suppressive genes in cancer biology [5]. For example, the tumor suppressive role of miR-625 has been widely explored. Decreased expression level of miR-625 is found in breast cancer [6], melanoma [7], and glioma [8]. But the functional role of this miRNA in LSCC remains largely elusive.

In the present study, we aimed to examine the expression profile of miR-625 in LSCC tissues and cell lines, evaluate the biological functions of miR-625 in LSCC cells, and identify the downstream target gene of miR-625 in LSCC. We believed that our findings might open new avenues for the treatment of this malignant disease.

## Materials and methods

### Patients and tissue samples

86 pairs of LSCC tissues and adjacent normal tissues (at least 1 cm from the neoplastic edge) were collected from LSCC patients who underwent partial or total laryngectomy at Affiliated Hospital of Hangzhou Normal University (Hangzhou, China) between March 2017 and May 2018. All recruited patients did not receive chemotherapy or radiotherapy preoperatively. The collected tissue samples were confirmed histologically by two experienced pathologists, snap-frozen in liquid nitrogen, and stored at −80°C. The research protocol was approved by the Ethics Committee of Affiliated Hospital of Hangzhou Normal University, and written informed consent was obtained from all patients or their relatives. The clinicopathological characteristics of LSCC patients are recorded in Table 1.

**Table 1:** Association between miR-625 expression level and clinicopathological characteristics of LSCC patients

Characteristics	Total number	Low expression (*n*=42)	High expression (*n*=44)	*P* -value
Age				0.174
<60	35	14	21	
≥60	51	28	23	
Gender				0.310
Male	59	31	28	
Female	27	11	16	
Smoking history				0.286
Yes	40	22	18	
No	46	20	26	
Differentiation				0.130
Well	56	24	32	
Moderately/poorly	30	18	12	
Lymph node metastasis				0.032
Yes	37	23	14	
No	49	19	30	
Clinical stage				0.010
I–II	47	17	30	
III–IV	39	25	14	

### Cell culture and transfection

LSCC cell lines (AMC-HN-8 and Tu-177), normal human keratinocyte (HaCaT), and human embryonic kidney cell line (HEK293T) were purchased from American Type Culture Collection (Manassas, VA, U.S.A.). Cells were cultured in Dulbecco’s modified Eagle’s medium (DMEM; Invitrogen, Carlsbad, CA, U.S.A.) containing 10% fetal bovine serum (FBS; HyClone, Logan, UT, U.S.A.), 100 U/ml penicillin, and 100 mg/ml streptomycin at 37°C in a humidified atmosphere with 5% CO_2_.

Synthetic miR-625 mimics (5′-AGGGGGAAAGUUCUAUAGUCC-3′) and mimics negative control (5′-CAGUACUUUUGUGUAGUACAA-3′) were obtained from Guangzhou Ribobio Co., Ltd (Guangzhou, China). The SOX4 overexpression plasmid was established by inserting the full-length CDS sequence of SOX4 into the pcDNA3.1 vector (Invitrogen). An empty vector was considered as a negative control. Cells were seeded in six-well plates at 80% confluence, and transfected with the plasmids and oligonucleotides using Lipofectamine 2000 (Invitrogen). After 48 h, the transfection efficiency was validated by RT-qPCR analysis.

### RNA isolation and RT-qPCR analysis

The total RNA from tissues or cells was isolated using Trizol Reagent (Invitrogen). Complementary DNA (cDNA) was generated using the PrimeScript RT reagent Kit (TaKaRa, Dalian, China), and PCR amplification was then performed using the SYBR Premix Ex Taq™ II kit (TaKaRa) on an ABI 7900 system (Applied Biosystems, Foster City, CA, U.S.A.). The relative expression levels of miR-625 or SOX4 mRNA were calculated using the 2^−ΔΔCt^ method [9], with U6 or GAPDH as the internal control. The primers were designed as follows: miR-625, 5′-GTCGTATCCAGTGCAGGGTCCGAGGTATTCGCACTGGATACGACGGACTA-3′ (RT), 5′-GCAGGGGGAAAGTTCTA-3′ (forward), and 5′-GTGCAGGGTCCGAGGT-3′ (reverse); U6, 5′-AACGCTTCACGAATTTGCGT-3′ (RT), 5′-CTCGCTTCGGCAGCACA-3′ (forward), and 5′-AACGCTTCACGAATTTGCGT-3′ (reverse); SOX4, 5′-CTTGACATGATTAGCTGGCATGATT-3′ (forward), and 5′-CCTGTGCAATATGCCGTGTAGA-3′ (reverse); GAPDH, 5′-CGACTTATACATGGCCTTA-3′ (forward) and 5′-TTCCGATCACTGTTGGAAT-3′ (reverse).

### Western blot analysis

Cells were lysed using ice-cold radio immunoprecipitation assay (RIPA) lysis buffer (Beyotime, Shanghai, China), and the protein concentration was measured using a BCA Protein Assay Kit (Solarbio, Beijing, China). Equal amounts of protein were fractionated by SDS-PAGE gel and then transferred onto polyvinylidene difluoride membranes (Millipore, Billerica, MA, U.S.A.). After blocking with 5% skim milk, the membranes were incubated overnight at 4°C with specific primary antibodies against SOX4 (1:1000; Santa Cruz Biotechnology, Inc., Dallas, TX, U.S.A.), E-cadherin (1:1000; Abcam, Cambridge, U.K.), N-cadherin (1:1000; Abcam), Vimentin (1:1000; Abcam), and GAPDH (1:1000; Santa Cruz Biotechnology, Inc.). After rinsing, the membranes were incubated with horseradish peroxidase-conjugated secondary antibodies for 1 h at room temperature. The signals were visualized using an ECL western blotting kit (Amersham Biosciences, Piscataway, NJ, U.S.A.), and GAPDH was set as the internal control.

## MTT assay

Cell proliferation was detected using (3-(4,5-dimethyl-thiazol-2-y1) 2,5-diphenyl tetrazolium bromide) (MTT) assay. Cells were seeded into 96-well plates at the density of 5 × 10^3^ cells/well and cultured for 24, 48, 72, or 96 h. Then 20 µl MTT (5 mg/ml; Sigma-Aldrich, St. Louis, MO, U.S.A.) was added to each well, and the plates were incubated for additional 4 h. After this, the medium was removed and 150  μl DMSO (Sigma-Aldrich) was added to each well. The absorbance of the solution was measured at 570 nm using a microplate reader (MultiskanEX, Lab systems, Helsinki, Finland).

### Colony formation assay

Cells were seeded on six-well plates at a density of 500 cells/well. The culture medium was replaced every 3 days. Ten days later, the colonies were fixed with 4% paraformaldehyde, stained with 0.1% crystal violet, and counted.

### Wound healing assay

Cells were seeded into 12-well plate and grown until 90% confluent. The cellular monolayer was then wounded using a sterilized 200 μl pipette tip, and then the cells were cultured in serum-free medium. Images were captured at 0 and 24 h following the initial scratch under an optical microscope.

### Transwell invasion assay

Cells were suspended in 200 ml of serum-free medium and placed in the upper chamber of the transwell filters (8 μm pore size; BD Biosciences, San Jose, CA, U.S.A.) that were coated with Matrigel (BD Biosciences). The lower chamber was filled with 600 µl medium containing 10% FBS as a chemoattractant. Following incubation for 24 h, the cells remaining on the upper side of the membrane were wiped off with cotton swabs, and the cells that moved to the bottom surface were fixed with 4% paraformaldehyde and stained with 0.1% crystal violet. The number of invaded cells was counted randomly in five fields of each membrane.

### Dual-luciferase reporter assay

The fragment from SOX4 3′-UTR containing the predicted miR-625 binding site was amplified by PCR and cloned into the psiCHECK2 vector (Promega, Madison, WI, U.S.A.). HEK293T cells were cultured in 24-well plates and co-transfected with 400 ng of luciferase reporter vectors comprising SOX4-WT or SOX4-MUT, 50 nmol/l of miR-625 mimics or mimics control, and 50 ng of pRL-TK plasmid (Promega) using Lipofectamine 2000. The pRL-TK Renilla luciferase plasmid was used as internal control. Forty eight hours after transfection, the luciferase activities were measured using the Dual-Luciferase Reporter Assay System (Promega), and the firefly luciferase activity was normalized to the Renilla luciferase activity.

## Statistical analysis

All statistical analyses were conducted using the GraphPad Prism 6.0 (GraphPad Software, Inc., La Jolla, CA, U.S.A.) and SPSS 17.0 (SPSS, Inc., Chicago, IL, U.S.A.). Differences between experimental groups were assessed by Student’s *t*-test or one-way analysis of variance (ANOVA). The association between miR-625 expression and clinicopathological characteristics of LSCC patients was evaluated using the chi-square test. All *P*-values were two-sided, and *P*<0.05 was considered statistically significant.

## Results

### miR-625 is down-regulated in LSCC tissues and cell lines

First, remarkably lower miR-625 expression was observed in LSCC tissues than that in the adjacent normal tissues (Figure 1A). In addition, the expression levels of miR-625 in the LSCC cell lines (AMC-HN-8 and Tu-177) were also significantly decreased compared with normal HaCaT cells (Figure 1B).

**Figure 1:** miR-625 is down-regulated in LSCC tissues and cell lines (**A**) RT-qPCR analysis of miR-625 expression levels in 86 pairs of LSCC tissues and adjacent normal tissues. (**B**) RT-qPCR analysis of miR-625 expression levels in LSCC cell lines (AMC-HN-8 and Tu-177) and normal HaCaT cells. *P<0.05 vs. HaCaT cells.

According to the average value of miR-625 expression, the LSCC patients were divided into high expression group (*n*=44) and low expression group (*n*=42). As listed in Table 1, low miR-625 expression was distinctly associated with advanced clinical stage (*P*=0.010) and lymph node metastasis (*P*=0.032) of LSCC patients.

### miR-625 inhibits LSCC cell proliferation

To further investigate the regulatory role of miR-625 in LSCC, we then transfected the LSCC cell lines (AMC-HN-8 and Tu-177 cells) with miR-625 mimics, and the ectopic expression of miR-625 was validated by RT-qPCR analysis (Figure 2A). The growth curves determined by MTT assay demonstrated that the proliferation abilities of AMC-HN-8 and Tu-177 cells were significantly impaired when miR-625 was overexpressed (Figure 2B). Besides, as demonstrated in Figure 2C, miR-625 overexpression also remarkably reduced the number of colonies formed by AMC-HN-8 and Tu-177 cells.

**Figure 2:** miR-625 inhibits LSCC cell proliferation (**A**) RT-qPCR analysis of miR-625 expression levels in AMC-HN-8 and Tu-177 cells after transfection. (**B**) The proliferation of AMC-HN-8 and Tu-177 cells after transfection was detected by MTT assay. (**C**) The clonogenic growth of AMC-HN-8 and Tu-177 cells after transfection was detected by colony formation assay. *P<0.05 vs. mimics control-transfected cells.

### miR-625 inhibits LSCC cell migration and invasion

Through wound healing assay, we found that the migratory abilities of AMC-HN-8 and Tu-177 cells were significantly inhibited by miR-625 overexpression (Figure 3A). We also performed transwell assay to examine cell invasive ability, and as shown in Figure 3B, miR-625 overexpression remarkably reduced the number of invaded AMC-HN-8 and Tu-177 cells.

**Figure 3:** miR-625 inhibits LSCC cell migration and invasion (**A**) The migration of AMC-HN-8 and Tu-177 cells after transfection was detected by wound healing assay. (**B**) The invasion of AMC-HN-8 and Tu-177 cells after transfection was detected by transwell invasion assay. (**C**) Western blot analysis of EMT-related protein expression levels in AMC-HN-8 and Tu-177 cells after transfection. *P<0.05 vs. mimics control-transfected cells.

EMT is a key event in cancer metastasis. As shown in Figure 3C, E-cadherin expression was significantly increased while the expression levels of N-cadherin and Vimentin were remarkably decreased in AMC-HN-8 and Tu-177 cells when miR*-*625 was overexpressed.

### miR-625 directly targets SOX4 in LSCC cells

To gain further insights into the functional role of miR-625 in LSCC, we then searched for its target genes. Through TargetScan website (http://www.targetscan.org) [10], we found that SOX4 3′-UTR contains a complimentary binding site of miR-625 (Figure 4A). In order to further confirm the prediction, we then performed dual-luciferase reporter assay. The results showed that miR-625 mimics significantly reduced the luciferase activity driven by SOX4-WT in HEK293T cells, but had no obvious effect on the activity of SOX4-MUT (Figure 4B). We further found that overexpression of miR*-*625 significantly decreased the protein expression levels of SOX4 in AMC-HN-8 and Tu-177 cells (Figure 4C). Furthermore, in LSCC tissues, remarkably higher SOX4 mRNA expression was observed (Figure 4D), and Pearson correlation analysis indicated that the expression levels of miR-625 and SOX4 mRNA were negatively correlated in LSCC tissues (*r* = −0.24, *P*=0.026; Figure 4E).

**Figure 4:** miR-625 directly targets SOX4 in LSCC cells (**A**) Sequences of the miR-625-binding sites in the human SOX4 3′-UTR. (**B**) Dual-luciferase reporter assay was performed to validate the between miR-625 and SOX4 3′-UTR. (**C**) Western blot analysis of SOX4 protein expression levels in AMC-HN-8 and Tu-177 cells after transfection. *P<0.05 vs. mimics control-transfected cells. (**D**) RT-qPCR analysis of SOX4 mRNA expression levels in 86 pairs of LSCC tissues and adjacent normal tissues. (**E**) Pearson correlation analysis of miR-625 and SOX4 mRNA expression levels in LSCC tissues.

### SOX4 blocks the tumor suppressive role of miR-625 in LSCC cells

Then we analyzed whether miR-625 inhibited the migratory and invasive capacities of LSCC cells partly by negative regulation of SOX4. As shown in Figure 5A, SOX4 overexpression rescued the impaired EMT in miR-625 mimics-transfected AMC-HN-8 and Tu-177 cells. Moreover, we also uncovered that SOX4 overexpression remarkably abrogated the inhibitory role of miR-625 on the migration and invasion of AMC-HN-8 and Tu-177 cells (Figure 5B,C).

**Figure 5:** SOX4 blocks the tumor suppressive role of miR-625 in LSCC cells (**A**) Western blot analysis of EMT-related protein expression levels in AMC-HN-8 and Tu-177 cells after transfection. (**B**) The migration of AMC-HN-8 and Tu-177 cells after transfection was detected by wound healing assay. (**C**) The invasion of AMC-HN-8 and Tu-177 cells after transfection was detected by transwell invasion assay. *P<0.05 vs. empty vector-transfected cells.

## Discussion

Initiation and progression of cancer are often caused by an imbalance between oncogenes and tumor suppressive genes. From The Cancer Genome Atlas (TCGA) database, a number of differentially expressed miRNAs in LSCC have been identified [11]. Several miRNAs, including miR-26a and miR-153, emerged as powerful regulators in LSCC, as indicated in recent studies [12,13]. One major finding of our study is that miR-625 was markedly decreased in LSCC tissue specimens and cell lines. Besides, decreased expression of miR-625 was associated with adverse clinicopathologic features of LSCC patients. In line with our clinical results, the *in vitro* experimental data also revealed that the ectopic expression of miR-625 led to the inhibition of LSCC cell proliferation, migration, and invasion. These results clearly implied that miR-625 may function as a tumor suppressor in LSCC.

Local invasion and distant metastasis are the main causes of death in LSCC patients [14]. EMT is a complex trans-differentiation process by which cancer cells gain migratory and invasion abilities [15]. We observed that miR-625 overexpression inhibited EMT in LSCC cells by increasing the expression levels of E-cadherin and decreasing the expression levels of N-cadherin and Vimentin. A miRNA can modulate a large number of target genes [16]. We then predicted the target gene of miR-625 using bioinformatics analysis and considered SOX4 as a potential target gene in LSCC. Sex-determining region Y-box 4 (SOX4), a master regulator of EMT, serves a fundamental role in tumorigenesis and metastasis [17,18]. Further rescue experiments confirmed that the tumor suppressive role of miR-625 in LSCC cells can be partly blocked by introduction of SOX4. Our data established a mechanistic link between miR-625, SOX4, EMT, and tumor metastasis.

Taken together, for the first time, we provided evidence that miR-625 is frequently down-regulated in LSCC and inhibits LSCC cell migration and invasion by targeting SOX4. Although the underlying mechanisms remain to be further elucidated, miR-625 may have potential application in miRNA-based therapy for LSCC patients in the future.

## Abbreviations

DMEM: Dulbecco’s modified Eagle’s medium
EMT: epithelial-mesenchymal transition
FBS: fetal bovine serum
LSCC: laryngeal squamous cell carcinoma
SOX4: Sex-determining region Y-box 4
